# Monitoring and Sharing of Music Teaching Environment Resources Using Big Data Technology

**DOI:** 10.1155/2022/3949443

**Published:** 2022-10-08

**Authors:** Caifen Yang

**Affiliations:** ^1^Northwest Normal University, Lanzhou, 730070, China; ^2^Lanzhou No.2 Middle School, Lanzhou, 730030, China

## Abstract

The teaching materials for different music courses in schools are getting more and more plentiful as education continues to become more and more digitised. This paper develops a resource monitoring and recommendation algorithm for the music teaching environment based on big data analysis technology, achieves the unified management and parallel retrieval of large music teaching resources, and completes the construction and sharing of music teaching resources with the goal of promoting online music teaching courses and increasing the efficiency of instruction. According to the experimental findings, the algorithm's recall and precision may both approach 95.84% and 95.19%, respectively. This demonstrates the benefits of this strategy. With the ability to analyse and retrieve large teaching resources and data quickly and accurately, this model can offer an advantageous solution for the storage and sharing of existing and future massive teaching resources. In order to effectively integrate music curriculum materials into our lessons, music teachers need to have a thorough awareness of not just the knowledge found in textbooks but also the adaptable use of music resources both within and outside of the classroom.

## 1. Introduction

With the expansion of business and culture, the country's education has also achieved rapid development. There are many different types of music curricular resources, and the extensive Internet platform offers a wealth of useful information for their integration. Network resources for music education span a variety of subject areas, demonstrating its breadth and depth while also having the potential to disseminate cutting-edge concepts and methods for music instruction [1]. The first step in providing individualised service is to have a thorough understanding of the needs of the learners, and the second is to create a learner-centered learning support system [2]. Despite having its benefits and merits in the modern network environment, particularly in the era of mobile Internet, traditional face-to-face instruction has not been able to keep up with the demands of students' learning and educational reform [3]. The network's benefits and education's deep integration with technology make it possible for those who need to learn to do so more conveniently, while also accelerating the updating of knowledge resources and fostering a comfortable learning environment for the advancement of knowledge literacy among all people.

The limitations of time and space can be removed from music instruction resources with the aid of the Internet [4]. Learning is everywhere if you want it to be, and online education offers students more practical and adaptable learning techniques. Each student's learning interest and learning ability will be different, so the page layout can be realized by using the frequency of students' online learning and the distribution of key points and difficulties [5]. Teachers or students typically use the traditional techniques of gathering resource data in the field of education, and information is found through scanning the internet or other media. We will fully utilise student academic records, browsing habits, internet records, and other data using DM (data mining) technology [6] to gather students' personality traits and transform teachers' educational expertise into rules and techniques that computers can follow. This work develops a recommendation algorithm for music instructional resources based on big data technology [7], achieves unified administration and parallel retrieval of enormous music instructional resources, and completes the creation and distribution of music instructional resources.

Educational big data is the core of constructing personalized instructional system [8]. Education covers a large number of people, and a large amount of data is produced all the time. The emergence of educational big data has created conditions for continuous innovation in the field of education, which has fundamentally changed the previous instructional mode, and finally provided the most suitable personalized education for each student [9]. The network's benefits and education's deep integration with technology make it possible for those who need to learn to do so more conveniently, while also accelerating the updating of knowledge resources and fostering a comfortable learning environment for the advancement of knowledge literacy among all people.

This research develops a sharing model of music education resources based on big data technology. Its key innovation is found in the following: (1) This paper integrates the student model with the instructional resource strategy, analyzes the characteristic information of learners by using DM technology, and grasps the learning status and cognitive level of each learner. (2) The model collects and analyzes the learners' recent usage information, analyzes the users' learning similarities, compares these data with DM patterns, and then sorts them according to the matching degree to predict the users' next learning content. (3) The model builds data for each user's learning records and analyzes their personal preferences and usage characteristics in combination with the basic information of users, so as to provide personalized services for learners in the music instructional environment.

## 2. Related Work

Individualized teaching has a strong realistic demand for innovative exploration of the future educational model. Extensive network music resources have greatly changed the traditional music teaching and also enriched the connotation of the traditional music teaching. School music education activities have made positive innovations in content organization and instructional development. Therefore, it is an urgent task for music educators in the information age to combine the development trend of information technology to promote the construction of online music education resources.

Maimaiti believes that using the Internet for online education has become the only way for modern education reform, and it is a good model to use the DM method to obtain the laws that exist between the data in the online instructional platform [10]. Qin believes that every user who participates in personalized learning can choose appropriate content according to their own interests, and through personalized push, anyone in the system can obtain learning content that suits their personal interests [11]. Pop et al. believe that some information in online teaching can be extracted by means of DM to form an optional data set that can be manipulated. By continuously enriching the data set, a more representative big data group can be formed, thereby providing better online education data support [12, 13]. Rickels et al. believe that higher education pays more attention to the quality of teaching, but there is still a certain lag in the improvement of online instructional platforms commonly used in higher education [14]. Wang believes that meaningful knowledge and potentially useful patterns extracted from DM can help improve education quality and student performance [15]. Deng and Dai pointed out that DM technology can not only be used in computer network instructional system but also can use web technology and mobile network technology to link with students' mobile terminals to obtain relevant information of students' learning data on mobile terminals [16]. Liang believes that the current is an era of data explosion. In this era, WEB-DM can be used to obtain relevant data, and then the improvement and secondary design of distance education platforms can reflect the characteristics of targeted learning programs [17].

The traditional educational resource system, which is centred on the system itself, does not fully take into account users' needs and habits, requires people to adapt to the system rather than the system adapting to users, and does not fully push according to people's individuality, which results in many issues like poor interactivity and low resource utilisation rate. In order to provide customised services for students in the music instructional environment, this study integrates the student model with instructional resources and methods and accomplishes unified administration and parallel retrieval of huge music instructional resources based on big data technology.

## 3. Methodology

### 3.1. Related Theoretical and Technical Basis

The data reflects the law, and the law guides the teaching [18]. This idea is one of the core ideas of using big data to guide education and teaching. Modern educational researchers explore the inherent laws among variables of all parties involved in education by developing DM models in different educational fields and then refine the laws for feedback guidance, which is convenient for educational decision-makers to plan and predict the overall trend and development prospects of education [19, 20]. In essence, DM technology is a technology that uses statistics to process database information. Its main purpose is to use data regularization to make it appear as quantitative and visualized available data. The main distinction between DM and traditional data analysis is that DM searches for knowledge and information without making firm assumptions. The data gathered by DM should have three qualities: it should be novel, efficient, and useful. Web mining is the process of using the DM principles and ideas to expand and improve existing mining techniques and apply them to Web information in order to mine and gather meaningful knowledge while focusing on the peculiarities of web information. It specifically means identifying intriguing, perhaps practical, and implicit patterns from a sizable number of web pages and web activity. The following is a brief summary of the general DM process: selection of the mining object, data preparation, modelling, DM, output of results, application of rules, etc. The typical DM process can be boiled down into three parts for practical purposes: (1) data preparation stage; (2) DM; and (3) output of results and consistent application. The rules that DM discovers are dynamic and only accurately reflect the rules of the most recent database. The database has to be updated whenever new information is added. Utilising educational big data to its fullest extent to draw on the traits of the educated can greatly aid in supporting personalized teaching and learning and make it possible to instruct pupils according to their ability.

The term “instructional resources” refers to the grouping of all instructional components that are based on learning objectives, implemented around learning activities, and created and applied to enhance learning quality and maximise learning activities [21]. From a connotation standpoint, instructional resources have the qualities of dynamic development, equal emphasis on learning and teaching, openness, and sharing under the combination of traditional instructional resources and information technology environment. It has created a network and divergent knowledge system through multimedia and network technology, and by combining these two in a particular method and with a person's preferences, it may enhance the effectiveness and standard of teaching and learning. The need for and conflict with sharing digital educational resources are currently becoming more and more obvious. How to swiftly locate the highest calibre resources in colleges and universities, how to successfully resolve all types of inconsistencies in the sharing process, and how to better popularise and distribute digital music instructional resources in colleges and universities, all of these require methodical, in-depth study and practise [22]. Digital music curriculum is an important part of music education resources. Accordingly, the development of digital music curriculum also occupies a very important position in the construction of music resources. Digital music curriculum can effectively solve the problem that traditional music education is confined to one place, and teachers and curriculum resources are relatively limited and can enable music learners and lovers in different regions to receive high-quality music education through the network. Constructing an open and interactive instructional resource sharing platform can realize the unification and integration of instructional resources, narrow the difference of instructional level caused by economic development and overall planning, promote the integration of resources between different regions, urban, and rural areas and schools, effectively promote the transformation of school education, teaching, management methods, and students' learning, and provide strong support for the transformation and development of education and teaching. The system structure of music course instructional resources is shown in Figure 1.

Each student can share resources, utilise teacher resources to the fullest extent, utilise his understanding of information technology, fully express his imagination, produce music, and gain the most learning from his successes by utilising the music course instructional resource system. The principles followed in the design of this system are as follows: (1) hierarchical design principle; (2) modular design principle; (3) principle of simplicity; and (4) the principle of extensibility. In the music course instructional resource system constructed in this paper, the courseware database is the main part of the instructional resource database. When teachers organize lesson plans, they need to take the courseware in the courseware database as the main body and organize and expand it into teaching courseware suitable for this course.

### 3.2. The Construction of Music Instructional Resource System

Users are the central component of the system-building process, and users are the source of the system's demand. As a result, user analysis comes first. The primary users of the music instructional resource system are students and teachers. There is a significant disparity in the system's operational level since students' operational levels are uneven, and teachers' majors are diverse. Therefore, it is essential to increase the system's usability and user friendliness when designing the system interface. Data must be processed and integrated before entering the data warehouse since the data inside is subject-oriented rather than application-oriented. There is a lot of historical data in the data warehouse that cannot be updated. At the same time, the data in the data warehouse changes with time, adding new data and deleting old data. Data warehouse needs to extract and prepare students' data, so as to significantly speed up DM. In this paper, the special markup function of XML language is used to standardize the description of irregular music education resources with small granularity, so that it has a unified metadata structure format. Based on this, the music education resources in the resource bank can be structured in an orderly way, and the education resource bank itself can also establish an efficient retrieval mechanism based on this, so as to provide the music education resources that meet the retrieval conditions of users more timely and accurately. At the same time, students can preview and deepen new knowledge points by watching the texts uploaded by teachers, microlessons, and other resources, so as to facilitate the understanding of new knowledge in class. User clustering needs an algorithm to calculate the initial cluster, but different algorithms have different advantages and disadvantages. Although the standard differential evolution algorithm has good global optimization ability, it also has obvious shortcomings. For example, the convergence speed of the algorithm is slow in the later stage of operation, so it cannot quickly converge to the optimal solution of the problem in less iterations. At the same time, the algorithm is very sensitive to the values of contraction factor and cross-over probability, and the settings of contraction factor and cross-over probability are often different for different problems. In this paper, the standard differential evolution algorithm is improved. To some extent, the improvement in this paper can make the original population conduct self-global fusion before global search and automatically mutate and screen to generate better population individuals, which effectively reduces the convergence speed of the previous algorithm, but the overall convergence speed is basically unchanged.

The knowledge network is a directed acyclic graph, because the degree of correlation between knowledge points is not the same, so in the graph, this paper sets a weight for each edge to represent the support strength between knowledge points. This paper uses a matrix to store the knowledge network. In a directed acyclic network *G*, if

(1) $$\begin{array}{c} e=\left(v_{i},v_{j}\right) \end{array}$$

exists, then *v*_*i*_ is called the premise node of *v*_*j*_; *v*_*j*_ is called the successor node of *v*_*i*_. The set of all prerequisite nodes of node *v* is denoted as Prenodes(v); the set of all subsequent nodes is Nextnodes(v). Then

(2) $$\begin{array}{c} \text{Prenodes}\left(\text{v}\right)=\left\{{\text{v}}_{\text{i}}\left|\left(v_{i},v\right)\in V\right.\right\}, \end{array}$$

(3) $$\begin{array}{c} \text{Nextnodes}\left(\text{v}\right)=\left\{v_{j}\left|\left(v_{j},v\right)\in V\right.\right\}. \end{array}$$

If

(4) $$\begin{array}{c} \left|\text{Prenodes}\left(\text{v}\right)\right|=0, \end{array}$$

then *v* is called the starting node, if

(5) $$\begin{array}{c} \left|\text{Nextnodes}\left(\text{v}\right)\right|=0. \end{array}$$

Then, *v* is called the terminal node. Nodes that are neither start nor end nodes are intermediate nodes. The set of all pre- and successor nodes of node *v* is called the neighborhood *δ*(*v*) of node *v*:

(6) $$\begin{array}{c} \delta \left(v\right)=\text{Pr}enodes\left(v\right)\cup Nextnodes\left(v\right). \end{array}$$

*TF* − *IDF* (term frequency-inverse document frequency) is a weighting method that is frequently used in data mining and information retrieval, figured out as follows:

Calculate word frequency:

(7) $$\begin{array}{c} TF=\frac{\text{The number of times a word appears in the text}}{\text{The total number of times in the text}}. \end{array}$$

A corpus that replicates the context in which the language is used is required to determine the inverse document frequency:

(8) $$\begin{array}{c} IDF=\log\left(\frac{\text{The total number of documents in the corpus}}{\text{The total number of documents containing the word}+1}\right). \end{array}$$

Calculate *TF* − *IDF*:

(9) $$\begin{array}{c} TF-IDF=TF\times IDF. \end{array}$$

In order to generate the set of frequent *k* itemsets constituting the set *L*_*k*_, a set of potential frequent *k* itemsets is generated in advance. If

(10) $$\begin{array}{c} p,q\in L_{k-1}, \end{array}$$

(11) $$\begin{array}{c} p=\left\{p_{1},p_{2},\cdots ,p_{k-2},p_{k-1}\right\}, \end{array}$$

(12) $$\begin{array}{c} q=\left\{q_{1},q_{2},\cdots ,q_{k-2},q_{k-1}\right\}, \end{array}$$

when 1 ≤ *i* ≤ *k* − 1, *p*_*i*_ = *q*_*i*_, when *i* = k − 1, *p*_*k*−1_ ≠ *q*_*k*−1_, then the following formula is the element in the set *C*_*k*_ of potential frequent *k* itemsets:

(13) $$\begin{array}{c} p\cup q=\left\{p_{1},p_{2},\cdots p_{k-2},p_{k-1},q_{k-1}\right\}. \end{array}$$

Crossing intermediate individuals in the original population and using the greedy strategy to choose the right data population before moving on to the next stage of screening the original population are the fundamental selection strategy of the original standard difference simplification algorithm in the calculation process. It can be described using the formula below:

(14) $$\begin{array}{c} X_{i}\left(g+1\right)=\left\{\begin{array}{c} U_{i}\left(g+1\right),\text{if f}\left[U_{i}\left(g+1\right)\right]\leq f\left[X_{i}\left(g\right)\right]\\ X_{i}\left(g\right),\text{other}. \end{array}\right. \end{array}$$

In the improvement process, this paper mainly optimizes the selection strategy. During the improvement process, the total 2*N* individuals in the original population *X*_*i*_(*g*) and population *U*_*i*_(*g* + 1) are rearranged according to their fitness; after the arrangement, only the first *N* individuals with the best adaptability are taken. A new population *W* is formed; then a new population *R* is obtained after another population mutation is performed using the above compilation operation.

In this paper, the instructional resource system of music course adopts the B/S architecture. The network topology diagram is shown in Figure 2.

There are two steps that must be taken to perfect the retrieval feature of the music education resource database. On the one hand, it is important to plan the progressive search feature or to set up advanced search on the foundation of primary search, so that consumers can perform secondary filtering on the search results. To effectively increase the retrieval range, however, we should develop the retrieval functionality of compound fields. In order to create the webpage of the database of music education resources, this work uses the XML language. From the viewpoint of the system, the entire system is divided into two parts: the portal website and background management, and the specific functional requirements are put into these two parts accordingly. This is done in order to reorganize the user requirements discovered through use cases and raise them to the height of the system. At the same time, by analyzing a large amount of information accumulated on the website, we can find patterns and rules that users are interested in and provide information for course designers and managers about improving course design and reconstructing the website, to provide teachers with information about students' learning courses and provide them with different learning contents according to their learning situation. In the use of resources, some resources are used frequently, and these resources can be regarded as high-quality resources. Generally speaking, high-quality resources are likely to be liked by all users, so the system will open up a special area on the main page and display it by resource ranking. Of course, users may also directly find the resources they want, and the system will provide the function of resource retrieval in a prominent position. Teachers can also upload their own resources in the way of knowledge tagging, so as to realize resource sharing. Because there are modules for browsing resources, managing resources, searching resources, system management, downloading tools, and so on, each module is aimed at different users. Therefore, according to the actual situation, according to the different levels of system users, different users are given permission control, which is divided into three levels of users: student users, teacher users, and system administrators. The modules that users of the three levels can access are different.

## 4. Result Analysis and Discussion

In this paper, the music course instructional resources in the form of distributed resources in the network are integrated and included, and a relatively complete resource index database is established in the local music education resource database, so that the number of its own resources is expanded and the quality is improved. The basic process of recommending resources for music course instructional resource system is as follows: firstly, determining the interaction process between students and the course system and accumulate information; using the accumulated information to establish a database; preprocessing the information data in the database; clustering users according to the processing results; carrying out similar matching on different clusters after clustering; and recommending courses according to the matching results. Music course instructional resource system consists of four servers. The specific allocation scheme is as follows: 1 application server, on which Tomcat is deployed; 1 name node acting as master, and 2 data nodes acting as slave.  Table 1 displays the test environment for this area.

The primary goal of the data preprocessing stage is to create a transaction database by cleaning, standardising, and integrating the data from user access logs and agent logs. Its goal is to compile the initial user logs left on the website into a data format that pattern mining algorithms for the DM stage may easily utilise. The algorithm is tested by Iris and Wine data sets. The basic experimental parameters are designed as follows: the scaling factor of standard differential evolution algorithm is 0.8, the cross-over probability is 0.9, and the population size is 20. The scaling factor of the improved differential evolution algorithm is 0.6-1.0, the cross-over probability is 0.7-1.0, and the threshold is 0.0001.  Figure 3 shows the training results of the algorithm.

Testing will be done on the processed data. The experimental findings are displayed in Table 2 as the average *F*-measure values of various algorithms on two data sets.

In order to discover the results matching keywords across several index files, resource retrieval involves using MapReduce. Naturally, the system will automatically create the index after the resource has been submitted. The primary retrieval algorithm is contained in the run () method of HadoopSearch when parallel retrieval is utilised. Following the retrieval, the system will order the retrieval results based on how closely the keywords were matched. First, this study conducts 10 experiments for each of the three indicators it has chosen: recall, precision, and similarity. The precision results of several algorithms are displayed in Figure 4. A comparison of recall rates for various algorithms is shown in Figure 5.

Recommend the relevant pages to the student users who access the system in accordance with the rules saved in the user feature database of the system and the sites that are currently being viewed. When a user first logs in, his feature library is empty, and the system does not suggest any pages to him. This document organizes the findings from six experiments into tables in order to more clearly depict the experimental outcomes of this strategy.  Table 3 displays the data outcomes for the indicators.

Firstly, the algorithm filters the user's conversation sequences and compares the length of each sequence in the latest conversation with the size of the active window. If the sequence length is less than or equal to the window size, keep the sequence unchanged. If the length of the sequence is larger than the window size, several pages in front of the sequence are cut off, and only the remaining pages with the last length equal to the window size are kept. At the same time, the algorithm evaluates the intermediate individuals, calculates the fitness, generates a new group according to the formula, and then continues to select the best individual for survival of the fittest.  Figure 6 shows the precision comparison of several algorithms.

The system creates a unified analysis data view to create a professional data warehouse using network teaching data as the primary data source, complemented by data from other information systems and external data sources. This system needs a particular level of dependability because it is designed with teachers and students in mind.  Figure 7 depicts the system's stability under heavy user traffic.

When numerous users access the system simultaneously, it is evident that its stability is still positive. This part evaluates the big data-based instructional resource system for music courses and examines the method suggested in this research. According to the experimental findings, this algorithm can achieve recall and precision of 95.84% and 95.19%, respectively. This demonstrates the benefits of this strategy. This system has produced the anticipated outcomes, is capable of integrating resources for music education successfully, and fulfils the goal of resource sharing.

## 5. Conclusion

The limitations of traditional music education in terms of time, place, and region have been overcome. Modern information technology has also increased the capacity and area of music education, greatly improved the means and resources for music instruction, expanded students' musical horizons, and made active, exploratory, and innovative learning possible for students. This research investigates the development and dissemination of big data-based music education materials. First, the concept, attributes, and importance of instructional resources are thoroughly examined in this paper. The relationship between instructional resources, instructional objectives, and instructional effects is theoretically analysed, as well as the crucial part that instructional resources play in students' learning and teachers' instruction. Then, a music course instructional resource system is constructed. The system collects and analyzes the recent usage information of learners, analyzes the learning similarities of users, compares these data with DM patterns, and then makes a specific ranking according to the matching degree, so as to predict the next learning content of users. Finally, this paper tests the music course instructional resource system and experiments the algorithm proposed in this paper. The experimental results show that the recall and precision of this algorithm can reach 95.84% and 95.19%, respectively. This shows that this method has certain advantages, and the system has achieved the expected results. It provides a beneficial solution for the storage and sharing of massive instructional resources and makes the analysis and retrieval of massive instructional resources and data fast and accurate. In the following stage, we will keep enhancing the big data-based functionalities of the music course instructional resource system and bring it even closer to the requirements of the application.

## Figures and Tables

**Figure 1:** System structure diagram.

**Figure 2:** System network topology diagram.

**Figure 3:** Training results of algorithm.

**Figure 4:** Comparison results of precision of algorithm.

**Figure 5:** Comparison results of recall rate of algorithm.

**Figure 6:** Accuracy comparison results of several algorithms.

**Figure 7:** Comparison of system stability.

**Table 1:** Test environment.

Testing environment	Set up
CPU	Dikaryon
Hard disc	2 TB
Network card	100/1000 self-adaption
Browser	IE
Development tools	Weka

**Table 2:** Average of *F*-measure of different algorithms on two data sets.

Algorithm	Iris data set	Wine data set
*K*-means algorithm	0.894	0.806
Association rule algorithm	0.885	0.824
Standard differential evolution algorithm	0.912	0.843
Improved algorithm in this paper	0.943	0.927

**Table 3:** Experimental results of different indexes.

Number of experiments	Recall ratio	Precision ratio	Similarity
1	93.31	95.19	0.135
2	92.89	93.42	0.127
3	95.08	95.02	0.162
4	93.24	94.97	0.148
5	94.78	92.18	0.139
6	95.84	94.86	0.140

## Data Availability

The data used to support the findings of this study are available from the corresponding author upon request.
